# Chemical Composition of Essential Oils of *Litsea cubeba* Harvested from Its Distribution Areas in China

**DOI:** 10.3390/molecules17067057

**Published:** 2012-06-08

**Authors:** Linlin Si, Yicun Chen, Xiaojiao Han, Zhiyong Zhan, Shengping Tian, Qinqin Cui, Yangdong Wang

**Affiliations:** 1 State key Laboratory of Forest Genetic and Tree Breeding, Chinese Academy of Forestry, Beijing 100091, China; 2 Institute of Subtropical Forestry, Chinese Academy of Forestry, Fuyang 311400, China; 3 College of Life Science, Anhui Agriculture University, Hefei 230036, China

**Keywords:** *Litsea cubeba*, essential oil, citral, D-limonene, varieties

## Abstract

*Litsea cubeba* (Lour.) Pers. is a promising industrial crop with fruits rich in essential oils. The chemical composition of essential oils of *L. cubeba* (EOLC) were determined for fruits harvested from eight regions in China. The overall essential oil content, obtained by hydrodistillation and analyzed by gas chromatography–mass spectrometry (GC-MS), ranged from 3.04% to 4.56%. In total, 59 compounds were identified, the dominant components being monoterpenes (94.4–98.4%), represented mainly by neral and geranial (78.7–87.4%). D-limonene was unexpectedly a lesser constituent (0.7–5.3%) in fruits, which differed from previous reports (6.0–14.6%). Several components were only detected in certain regions and compounds such as *o*-cymene and eremophilene have never before been reported in EOLC. These results demonstrate significant regional variation in the chemical composition of EOLC. This investigation provides important information with regard to the bioactivity, breeding work and industrial applications of *L. cubeba*.

## 1. Introduction

The genus *Litsea* (Lauraceae) is composed of ca. 622 species, distributed mainly in tropical and subtropical Australia, New Zealand, North America, South America, and Asia [1]. China alone has 74 species [2], among which *Litsea cubeba* (Lour.) Pers. is a perennial, dioecious tree or shrub, widespread in areas of southern China. 

Like other plants of the genus *Litsea*, *L. cubeba* produces an essential oil (EOLC), which can be extracted from different parts of the plant, including the fruit, root and flower as well as stem and leaf, with significant diversity in composition and yield [3,4]. EOLC is a flowing, pale yellow liquid, with an intensely lemonlike, spicy aroma [5]. It has been widely employed in the food, chemical and medicinal industries. In China, the Ministry of Health has approved EOLC for use as a food additive in accordance with standard GB 2760-2007. Furthermore, EOLC has been used as a crude material for the manufacture of citral, vitamins A, E, and K, ionine, methylionone, and perfumes [6]. Extracts of *L. cubeba* have also been used in traditional Chinese medicine for the treatment of a variety of ailments [7]. Recently reports have demonstrated the bioactivities of EOLC, which include antibacterial [8], antifungal [9,10], acaricidal [11], insecticidal [12,13], antioxidant [14], and anticancer properties [15]. 

The biological activities of EOLC are attributed directly to the synergistic or antagonistic effects of its chemical composition. Therefore, intimate knowledge of the chemical composition of EOLC is important for understanding its role in biological systems. Several researchers have reported the essential oil compositions of *L. cubeba* from limited geographical areas. Twenty components were isolated from EOLC harvested from Hunan Province [16]. Zhou and Mo [17] also identified 20 constituents in EOLC taken from Guizhou Province, and 31 compounds were identified in EOLC from Guanxi Province [18]. However, each of these studies applied their own sets of extraction and purification conditions. 

In general, the relative composition of essential oils varies remarkably with geographical position, climate conditions and several other factors [19]. To acquire more information, the current study determined the essential oil compositions of *L. cubeba* collected from different parts of China. This work lays a theoretical foundation for further pharmacological research to explore the properties of EOLC and provides a reference for later breeding of this plant. 

## 2. Results

Plants were sampled primarily from hills and barren lands. Climatic information for these areas is provided in Table 1. Most were subtropical zones marked by warm and humid climates. Fresh fruits of *L. cubeba* afforded yellowish oils, with yields (mean of four replicates) ranging from 3.14% (D) to 4.56% (G) by dry weight (see Figure 1). In total, 59 individual components (41 monoterpenes, 15 sesquiterpenes, and three non-terpene compounds) were isolated and identified. Retention indices, relative percentages, and methods used for identification are listed in Table 2.

**Table 1:** Climate and geographic habitats of *Litsea cubeba*.

	Latitude(°)	Longitude(°)	Elevation(m)	T _max_(°C)	T _min_(°C)	T _average_(°C)	Precipitation(mm)
A	27.15 N	118.27 E	609	40.7	−7.2	18.7	1662.9
B	25.97 N	117.41 E	495	39.8	−6.0	19.3	1563.8
C	25.23 N	115.30 E	271	40.0	−3.8	19.4	1461.2
D	27.39 N	114.35 E	260	39.9	−5.5	17.6	1643.6
E	27.35 N	105.43 E	1608	36.2	−10.9	12.7	899.5
F	26.34 N	111.80 E	137	39.7	−7.0	17.8	1425.7
G	24.42 N	100.74 E	2068	37.3	−1.4	18.6	1131.6
H	28.19 N	104.51 E	823	39.5	−1.7	17.8	1063.1

Elevation is given as an average: T_max_ = Annual extreme maximum temperature; T _min_ = Annual extreme minimum temperature; T_average_ = Annual average temperature; Precipitation = Annual precipitation. Locations of *L. cubeba*: A, B = Fujian Province; C, D = Jiangxi Province; E = Guizhou Province; F = Hunan Province; G = Yunnan Province; H = Sichuan Province.

**Figure 1:** Essential oil yields of *Litsea cubeba* harvested from different areas.

Of the monoterpene constituents, most were oxygenated, including 28 of the monoterpenes in oil A (97.4% of the total oil), 26 in oil B (98.4% of the oil), 30 in oil C (96.5% of the oil), 23 in oil D (97.3% of the oil), 28 in oil E (98.0% of the oil), 23 in oil F (98.4% of the oil), 20 in oil G (94.6% of the oil), and 26 in oil H (94.4% of the oil). The predominant compounds were neral and geranial, accounting for 78.7% (G) to 87.4% (E) of the total oil of *L. cubeba*. Note that, neral and geranial are* cis-trans* isomers of citral. Neral always occurred in higher quantities than geranial. The citral content in sample G was relatively low, despite a higher relative yield of oil.

**Table 2:** Essential oil compositions of *Litsea cubeba* harvested from different areas.

	Components	Peak area (%)									Identification ^b^
		RI ^a^	A	B	C	D	E	F	G	H	
1	α-Pinene	930	0.2	0.1	0.3	0.2	0.1	0.1	0.1	0.1	GC-MS,RI
2	Camphene	944	0.1	t ^c^	0.2	0.1	t	0.1		0.1	GC-MS,RI
3	β-Phellandrene	970	t	0.4	t	t	t	t	0.1		GC-MS,RI
4	β-Pinene	972	0.3	0.2	0.3	0.2	0.1	0.1	0.1	0.1	GC-MS,RI
5	Methyl heptenone	987	0.8	0.5	0.3	0.5	0.5	0.2	0.6	0.9	GC-MS,RI
6	2,3-Dehydro-1,8-cineole	989				t		0.1			GC-MS,RI
7	β-Myrcene	991	0.7	0.3	0.8	0.6	0.3	0.5	0.5	0.6	GC-MS,RI
8	2-Methyl-6-hepten-1-ol	995			t				0.1		GC-MS,RI
9	α-Phellandrene	1003	0.2		t						GC-MS,RI
10	3-Carene	1008							t		GC-MS,RI
11	α-Terpinene	1015		t							GC-MS,RI
12	p-Cymene	1020							t		GC-MS,RI
13	*o*-Cymene	1022	t								GC-MS,RI,RT
14	D-limonene	1026	5.0	2.5	5.3	4.1	0.7	3.1	1.3	2.4	GC-MS,RI,RT
15	Cineole	1028	0.4	0.4	0.2	0.4	0.1	0.3	0.2	0.1	GC-MS,RI
16	β-( *E*)-Ocimene	1038			t		0.1			t	GC-MS,RI
17	β-( *Z*)-Ocimene	1047	0.1		t		0.3			t	GC-MS,RI
18	γ-Terpinolene	1056		t							GC-MS,RI
19	( *Z*)-β-Terpineol	1066		t							GC-MS,RI
20	Terpinolene	1085	0.1	t	t		t			t	GC-MS,RI
21	(+)-4-Carene	1086				t		t			GC-MS,RI
22	Linalool	1101	1.5	1.5	1.2	1.3	1.3	1.4	1.4	1.6	GC-MS,RI
23	( *Z*)-Limonene oxide	1131			t					t	GC-MS,RI
24	( *E*)-Limonene oxide	1136			t		t			0.1	GC-MS,RI
25	Camphor	1140	t								GC-MS,RI
26	Isopulegol	1143				1.1	t		t		GC-MS,RI
27	Citronellal	1153	0.6	0.8	1.8		1.3	1.5	6.2	1.3	GC-MS,RI
28	Borneol	1163	0.2	0.1	0.2						GC-MS,RI
29	Verbenol	1165	1.4	1.2	1.4	1.4	1.3	1.3	1.5	1.8	GC-MS,RI
30	Terpinen-4-ol	1175	0.1	0.3	0.1	0.1	0.1	t		0.1	GC-MS,RI
31	Isopulegone	1183	2.1	1.8	1.9	2.1	1.8	1.9	2.0	2.5	GC-MS,RI
32	α-Terpineol	1189	0.4	0.4	0.2	0.4	0.1	0.4	0.2	0.2	GC-MS,RI
33	*cis*-Piperitol	1199	t				t				GC-MS,RI
34	*cis*-Carveol	1205	0.1	t	t	0.1	t	t		t	GC-MS,RI
35	( *S*)-Citronellol	1223			t		t				GC-MS,RI
36	Nerol	1230	0.8	1.3	0.5	0.6	1.0	0.2	0.9	0.7	GC-MS,RI
37	( *R*)-Citronellol	1233	0.1	0.2	0.3	0.2	0.3	0.2	0.8	0.5	GC-MS,RI
38	Isogeraniol	1237			t					t	GC-MS,RI
39	Neral	1245	35.7	36.3	34.7	35.7	37.4	37.0	34.2	35.4	GC-MS,RI,RT
40	Piperitone	1253	t	t	0.1	t	t	t	t	t	GC-MS,RI
41	Geraniol	1258	1.4	2.6	0.7	1.5	1.4	0.8	0.7	0.4	GC-MS,RI
42	Geranial	1276	45.9	48.0	45.9	47.2	50.0	49.5	44.4	46.2	GC-MS,RI,RT
43	Geranic acid	1359	0.1	t	0.2	0.1	0.2	t		0.2	GC-MS,RI
44	Copaene	1371			0.1					t	GC-MS,RI
45	Geranyl acetate	1384						t			GC-MS,RI
46	β-Elemene	1388			0.1	t		t			GC-MS,RI
47	β-Caryophyllene	1420	0.3	0.1	0.3	0.3	0.1	0.3	0.1	0.8	GC-MS,RI
48	β-Farnesene	1456					0.4		2.3	2.0	GC-MS,RI
49	α-Caryophyllene	1462	t		0.1	0.1	t	t		t	GC-MS,RI
50	Germacrene D	1485			t			t			GC-MS,RI
51	γ-Elemene	1496		t					t		GC-MS,RI
52	Eremophilene	1502						t			GC-MS,RI,RT
53	Germacrene A	1503			0.1	t					GC-MS,RI
54	β-Bisabolene	1510								t	GC-MS,RI
55	Cadinene	1526	t		0.1						GC-MS,RI
56	Caryophyllene oxide	1586	0.1	t	0.2	0.1	0.1	0.1	t	0.3	GC-MS,RI
57	Humulene epoxide II	1613								t	GC-MS,RI
58	Selina-6-en-4-ol	1624	t								GC-MS,RI
59	α-Cadinol	1662	t								GC-MS,RI
	Total compounds 59		35	30	40	29	33	31	26	34	
	Monoterpene hydrocarbons		6.6	3.5	7.0	5.2	1.6	3.9	2.1	3.3	
	Oxygenated monoterpenes		90.7	95.0	89.5	92.2	96.4	94.5	92.5	91.1	
	Sesquiterpene hydrocarbons		0.3	0.1	0.6	0.5	0.5	0.4	2.4	2.9	
	Oxygenated sesquiterpenes		0.1	t	0.2	0.1	0.1	0.1	t	0.3	
	Non-terpenes		0.8	0.5	0.3	0.5	0.5	0.2	0.7	0.9	
	Total identified		98.7	99.1	97.6	98.3	99.0	99.2	97.8	98.5	

^a^ Retention index on a Hewlett Packard 5MS column; ^b^ GC-MS = identification based on a high-quality match of mass spectra; RI = Retention index compared with those in the literature; RT = Retention time compared with authentic compounds; ^c^ t = Trace component (<0.1%). Sample location: A, B = Fujian Province, C, D = Jiangxi Province, E = Guizhou Province, F = Hunan Province, G = Yunnan Province, H = Sichuan Province.

The chemical compounds present in all of the oils were neral, geranial, α-pinene, β-pinene, methyl heptenone, β-myrcene, D-limonene, cineole, linalool, citronellal, verbenol, isopulegone, α-terpineol, (*R*)-citronellol, piperitone, geraniol, β-caryophyllene and caryophyllene oxide. D-limonene prevailed in the third oil extracted from *L. cubeba* samples A, C, D, F, but was substituted for geraniol, isopulegone, citronellal and isopulegone in the oils of samples B, E, G, and H, respectively. Other constituents were only identified in samples obtained from certain regions. These unique compounds included *o*-cymene, camphor, selina-6-en-4-ol, α-cadinol in oil A, α-terpinene, γ-terpinolene and (*Z*)-β-terpineol in oil B, geranyl acetate and eremophilene in oil F, 3-carene and *p*-cymene in oil G, and β-bisabolene and humulene epoxide II in oil H. Only trace amounts of these unique compounds were shared among samples.

## 3. Discussion

Unexpectedly, d-limonene was present in EOLC only as a minor constituent (0.7–5.3%), which differs significantly from the findings of previous studies [20,21,22], where it was a primary component (6.0–14.6%). In addition, certain trace compounds, such as *o*-cymene and eremophilene had never before been found in oil obtained from *L. cubeba* friut. *o*-Cymene has, however, been found in the leaf oil of *Litsea glutinosa* in trace amounts of less than 0.1% [23], and eremohpilene has been reported in other Lauraceae plants [24].

As expected, both quantitative and qualitative differences in composition were observed among the essential oils, all of which contained citral as the primary ingredient. Even EOLCs from the same province exhibited significant differences in composition. Even plants gathered at the same stage of development and from within the same locality and ecological environment have shown possible differences in their essential oils [25]. EOLC composition may ultimately result from gene-environment interactions.

EOLC is natural product, consisting primarily of terpenes with some non-terpene compounds. Terpenes were thought to be products of detoxification and overflow metabolism until several were confirmed to be repellents or attractants to other organisms. This led to the belief that terpenes play an important role in antagonistic or mutualistic interactions between organisms [26]. Synthesis-related enzyme genes of some terpenes in EOLC have been partially functionally characterized [27]. Nevertheless, we still know relatively little about their actual bioactivity. Biological activity can vary depending on the composition of the essential oil [28]. Therefore, the bioactivity of EOLC may depend on the area from which it is harvested.

Note that the current study examined the chemical compositins of *L. cubeba* oil taken from several provinces in China. Preliminary information does exist, however, on the chemical fingerprint of *L. cubeba* from those provinces and will be the focal point of a future study. The powerful tools provided by modern molecular biology, chemical biology, and analytical chemistry promise to yield a much more comprehensive view of the terpenes associated with bioactivity.

## 4. Experimental

### 4.1. Plant Materials

Aerial parts of *L. cubeba* were randomly collected in September 2011 from the plant’s natural habitat: Jianou and Yongan of Fujian Province (A, B), Anyuan and Fenyi of Jiangxi Province (C, D), Bijie of Guizhou Province (E), Yongzhou of Hunan Province (F), Jingdong of Yunnan Province (G) and Changning of Sichuan Province (H). Only fresh, mature, and healthy fruits were chosen as samples. All samples were transported immediately to the lab and air-dried at ambient temperature prior to essential oil extraction. The fruits of *L. cubeba* were authenticated morphologically and microscopically by Vice-Prof. Shengni Tian, Anhui Agriculture University, China. Voucher specimens have been deposited in the Herbarium of the College of Life Science, Anhui Agriculture University, China.

### 4.2. Chemicals and Reagents

All chemicals and reagents were of analytical grade. Standards were supplied by Sigma-Aldrich Company (Steinheim, Germany).

### 4.3. Isolation of Essential Oils

The dried vegetable matter (100 g) was subjected to hydrodistillation using a Clevenger-type apparatus to extract essential oil. The Clevenger-type apparatus consisted of a 2,000-mL flask, a vertical tube, a condenser, a measuring tube with stopcock, and a return tube. The return tube connected the bottom of the measuring tube to the vertical tube, which combined with the top of the condenser. The flask was filled with 1,500 mL of distilled water and heated by an electric heating mantle. The extraction time was 5 h, after which no more essential oil was obtained. The volatile distillate was dried over anhydrous sodium sulfate and stored at 4 °C until subsequent analysis.

### 4.4. GC-MS Analysis

GC-MS analysis was carried out on an Agilent 6890N gas chromatograph coupled to a mass spectrometer (Agilent 5975B, Santa Clara, CA, USA) using a fused silica capillary column (HP-5MS) coated with polydimethylsiloxane (19091 S-433) (30 m × 0.25 mm internal diameter, 0.25 μm film thickness). The column temperature was set at 50 °C for 2 min, ramped at a rate of 3 °C/min to 120 °C for 2 min, then increased to 250 °C at 15 °C/min for 5 min. Helium was used as the carrier gas at a flow rate of 1 mL/min. The sample was diluted in the ether (1:10) and a volume of 1.0 μL was injected. The injector was held at 220 °C and operated in the split mode at a ratio of 1:40 for each sample. The MS operating parameters were an ionization voltage of 70 eV, ion source temperature of 230 °C, and electron multiplier energy of 1,024 V.

### 4.5. Qualitative and Quantitative Analysis

Compound identifications were based on comparisons their mass spectra with the mass spectra obtained from a MS database (NIST 08) and by comparisons of the RI with values reported in the literature [29,30] or against values obtained on authentic compounds. A homologous series of *n*-alkanes (C_7_–C_30_) were run under the same operating conditions as the essential oil to determine RIs. The relative amounts of individual components were calculated via peak area normalization.

### 4.6. Data Analysis

Yields of essential oil are expressed as mean values ±1 standard deviation. Graphs were drawn in SigmaPlot v10.0. Images were identically processed using Adobe Photoshop CS5 software.

## 5. Conclusions

EOLCs harvested from various areas of China were obtained by hydrodistillation of *L. cubeba* and analyzed by GC-MS. Fifty-nine components were identified. Citral was the most abundant component in all of the oils. The relative composition of EOLC varied with the region from which the sample was collected. For the first time, eremophilene and *o*-cymene were identified in EOLC.
